# Assessment of Mental Workload by Visual Motor Activity among Control Group and Patient Suffering from Depressive Disorder

This article has been retracted.

**DOI:** 10.1155/2022/8555489

**Published:** 2022-03-31

**Authors:** G. Murugesan, Tousief Irshad Ahmed, Mohammad Shabaz, Jyoti Bhola, Batyrkhan Omarov, R. Swaminathan, F. Sammy, Sharmin Akter Sumi

**Affiliations:** ^1^Department of Computer Science and Engineering, St. Joseph's College of Engineering, Chennai 600119, India; ^2^Department of Clinical Biochemistry, Sher-i-Kashmir Institute of Medical Sciences, Soura, Srinagar, J&K, India; ^3^Model Institute of Engineering and Technology, Jammu, J&K, India; ^4^Electronics & Communication Engineering Department, National Institute of Technology, Hamirpur, India; ^5^Al-Farabi Kazakh National University, Almaty, Kazakhstan; ^6^International University of Tourism and Hospitality, Turkistan, Kazakhstan; ^7^Suleiman Demirel University, Kaskelen, Kazakhstan; ^8^Saveetha School of Engineering, Chennai, Tamil Nadu, India; ^9^Department of Information Technology, Dambi Dollo University, Dembi Dolo, Welega, Ethiopia; ^10^Department of Anatomy, Bangabandhu Sheikh Mujib Medical University, Dhaka, Bangladesh

## Abstract

Major depressive disorder (MDD) is a mood state that is not usually associated with vision problems. Recent research has found that the inhibitory neurotransmitter GABA levels in the occipital brain have dropped. *Aim*. The aim of the research is to evaluate mental workload by single channel electroencephalogram (EEG) approach through visual-motor activity and comparison of parameter among depressive disorder patient and in control group. *Method*. Two tests of a visual-motor task similar to reflect drawings were performed in this study to compare the visual information processing of patients with depression to that of a placebo group. The current study looks into the accuracy of monitoring cognitive burden with single-channel portable EEG equipment. *Results*. The alteration of frontal brain movement in reaction to fluctuations in cognitive burden stages generated through various vasomotor function was examined. By applying a computerised oculomotor activity analogous to reflector image diagram, we found that the complexity of the path to be drawn was more important than the real time required accomplishing the job in determining perceived difficulty in depressive disorder patients. The overall perceived difficulty of the exercise is positively linked with EEG activity measured from the motor cortex region at the start of every experiment test. The average rating for task completion for depression patients and in control group observed and no statistical significance association reported between rating scale and time spent on each trial (*p*=1.43) for control group while the normalised perceived difficulty rating had 0.512, 0.623, and 0.821 correlations with the length of the pathway, the integer of inclination in the pathway, and the time spent to complete every experiment test, respectively (*p* < 0.0001) among depression patients. The findings imply that alterations in comparative cognitive burden levels during an oculomotor activity considerably modify frontal EEG spectrum. *Conclusion*. Patients with depression perceived the optical illusion in the arrays as weaker, resulting in a little bigger disparity than individuals who were not diagnosed with depression. This discovery provided light on the prospect of adopting a user-friendly mobile EEG technology to assess mental workload in everyday life.

## 1. Introduction

The human cognitive system is of interest to researchers working on computational applications for a variety of reasons across many fields. For more than three decades, researchers have been seeking to overcome this challenge to understand human cognitive capability [1, 2]. In major depressive disorder, abnormalities in motor activity are linked to other characteristics such as a lack of interest in daily chores (MDD). As a consequence, patients with current MDD have lower motor activity [3, 4], and treatment response has been linked to increased motor activity [5, 6].

Here, we also brief about other mental illness disorders.

- Anxiety: unlike typical feelings of apprehension or anxiety, anxiety disorders are characterized by excessive fear or anxiety. The most common mental ailments are anxiety disorders. Anxiety sufferers may strive to avoid circumstances that aggravate or cause their symptoms. Workplace productivity, schoolwork, and personal relationships could all be harmed. Generalized anxiety disorder, panic disorder, particular phobias, agoraphobia, social anxiety disorder, and separation anxiety disorder are all examples of anxiety disorders.
- Panic disorder: the most prevalent symptom of panic disorder is recurrent panic attacks, which are characterized by an overwhelming combination of physical and psychological anguish. Many of these symptoms, such as trembling or shaking, palpitations, pounding heart or high heart rate, perspiration, feeling alienated, and fear of losing control, might occur simultaneously during an attack. [7].
- Posttraumatic stress disorder (PTSD): people who have been threatened with death, sexual violence, or serious injury, or who have experienced or witnessed a traumatic incident such as a natural disaster, a catastrophic accident, a terrorist attack, war/combat, or rape, may develop posttraumatic stress disorder (PTSD). People with PTSD have strong, unsettling thoughts and feelings about the traumatic event that last long after it has happened. They may have flashbacks or dreams about the event, as well as feelings of sadness, fear, or anger, as well as a sense of being distant or estranged from people [8].
- Dissociative Disorders: dissociative disorders impact memory, identity, emotion, perception, conduct, and sense of self. Dissociative symptoms can impact every element of a person's mental health. Detachment or feeling as if one is outside one's body, as well as memory loss or amnesia, are examples of dissociative symptoms. Dissociative illnesses are typically linked to traumatic experiences in the past [9].

Neuropsychological problems are common symptoms in people suffering from chronic fatigue syndrome (CFS). The goal of the study was to compare the cognitive abilities of CFS patients to those of two illness comparator groups (nonmelancholic depression and acute infection), as well as healthy controls [10, 11]. However, quantitative measurements of motor activity have become more common in recent years. On the one hand, miniaturized accelerative devices with great reliability and validity have been developed as a result of technological advancements [12]. Recall questionnaires, on the other hand, were found to have only limited validity in metaanalyses [13]. Women are diagnosed with depression at a higher incidence than men, which may be due to women's proclivity to seek treatment as soon as possible [14, 15]. In accordance with this, latest long-term telehealth strategies use objectively assessed cognitive movement as a replacement for depressed clinical signs.

The relationship between mental and physical health is mentioned here. Chronic physical illnesses get worsened by poor mental health. People who are suffering from major mental diseases are more likely to develop chronic physical ailments. Those patients who have severe physical disorders are more prone to develop mental problems [16, 17]. The connection among psychological and physical health is well established [18], While new technologies are being developed to observe numerous indices of physical health with wearable and wireless devices, such as pulse, blood pressure, and body temperature [19, 20], the alternatives for monitoring cognitive burden are far more limited. The difficulty of reliably measuring and quantifying mental states is one of the key obstacles.

A transportable EEG system with several functional prototypes has recently been suggested. The preponderance of these recommended mobile EEG devices offers consumers a wireless and feasible option for monitoring their real-time brain processes while maintaining the excellent transient response of data gathered by conventional laboratory EEG equipment [21]. Mobile electroencephalography (mobile EEG) is the next neuroscientific device for studying real-time activity in the brain that is fairly affordable, noninvasive, and has portability. It takes an advantage of cutting-edge hardware, as well as the long-established advantages of traditional EEG and recent signal processing advancements [22, 23]. The EEG signals obtained through such mobile equipment and applications have been convenient in assessing and determining the metal conditions of users [24]. As a result, the purpose of this study was to see if a single-channel dry sensor mobile EEG device could be used to assess cognitive burden. In addition to the conventional wet EEG system, which emerges with various tech challenges such as skin and electrode readiness, user discomforts, and lengthy preparation time, the dry sensor EEG system's ergonomic design and high flexibility enable us to evaluate the psychological condition of users during an unrestrained innate activity, in a physical world establishing well outside research lab.

In major depressive disorder (MDD), both quantitative and qualitative cognitive evaluations are changed, but there is minimal correlation between them especially in those with residual mood symptom everyday memory and related cognitive concerns expressed by people should prompt further research into sleep quality and (or) additional health related complications, as these conditions are known to impact mental enactment [25, 26]. Sleep, for instance, may have mental confusion, disorientation, or delirium effects [27], and the lack of good quality sleeping hours impacts a variety of cognitive domains [28]. Depression is not a natural element of getting older and should never be overlooked or neglected. Unfortunately, geriatric depression is commonly misunderstood and neglected, but they may be hesitant to seek treatment. A few of the depression symptoms in the elderly may differ or be less evident, which could be memory problems or personality shift aches, and aches all throughout the body [29, 30]. Although there is evidence that visual processing is disrupted in MDD, it is unclear whether the loss is in retinal or cortical processing (or both). A retinal deficiency would imply more localised alterations in visual information processing, whereas a cortical deficit could indicate a more general abnormality. Electrophysiological and behavioural examinations of contrast perception in major depressive disorder (MDD) have produced mixed results, and most previous behavioural research has examined contrast detection at the threshold. From a practical perspective, visual contrast tests are a quick, easy, and noninvasive procedure that could be refined further to serve as biomarkers for aberrant visual information processing in depression. This discovery provided light on the prospect of adopting a user-friendly mobile EEG technology to assess mental workload in everyday life.

### 1.1. Importance of the Study

Two of the most prevalent persistent problems among MDD patients who achieve clinical remission are cognitive dysfunction and functional impairments. Our findings include a mental workload assessment of MDD patients and a control group, as well as moderate impact sizes in the neurocognitive domains of processing speed, attention, executive function, learning, and memory.

### 1.2. Objective

The objective of the research is to evaluate mental workload by a single channel EEG approach, brain rhythms through visual-motor activity, and comparison of parameter among depressive disorder patient and in control group.

## 2. Method

### 2.1. Participants

For this investigation, a total of twenty participants were enrolled. Ten individuals have healthy or actually corrected eyesight and have never had a neurodegenerative or psychiatric problem. An average age of control group is 28.3 ± 3.2 years. While other ten participants have average age of 27.3 ± 2.8 years. The beck depression inventory (BDI) [28] was conducted before pretesting at a psychologist's institute, and these subjects were enrolled based on their results. For the depressive disorder patients, BDI score above 30 was considered (Table 1). The BDI toll was employed since it is a frequently used depression assessment measure in research and clinical practise. Participants with elevated levels of depression and nondepressed controls will be easily identified using this assessment. For validity and reliability, the BDI has been standardised in several countries and cultures [31, 32].

Ethical clearance: the data collecting format and experimental methodologies to prospectively acquire thorough information on acute stroke patients in order to conduct this study were approved by the Institutional Committee as well as a partner hospital. Each patient was required to complete an informed consent form. The entire data gathering procedure was carried out in compliance with the methodology and standards that had been accepted. On request, a full form will be provided.

Healthy individuals are administered through a phone screening session.

#### 2.1.1. Inclusion Criteria

Both control and depressive patients had to be highly right handed (a rating of 34 on Chapman & Chapman's 1987 39-point scale). Age was <18 years for both groups. For the depressive disorder patients, BDI score above 30 was considered.

#### 2.1.2. Exclusion Criteria

- For Control group: participants have no background of head injury with failure of consciousness lasting more than 10 minutes, cerebrovascular accident, seizure disorders, electroconvulsive therapy, usage existing psychiatric drugs, or frequent suicidal behaviour (though respondents with present mental and rehabilitation therapy were consider). The healthy controls had no current or prior history of mental illness, and they said that they had no relatives with Axis I disorders such as anxiety, panic disorder, dissociative disorders, or posttraumatic stress disorder.
- BDI score was >30, as well as other comorbid conditions and mental illnesses were acute suicidality, depressive disorder with psychotic symptoms, bipolar disorder, organic psychiatric disorders, substance-abuse disorders, schizophrenia, schizoaffective disorders, and borderline personality disorder for the depressive disorder group.

### 2.2. Data Trial

Ten trials of computerised visual motor activity were completed by all subjects. Milner was the first to utilise the mirror drawing challenge to see how cognitive deficits affected learning and developing motor skill [33]. In order to complete the tasks correctly, respondents were had to develop a unique set of visual-motor connections (i.e., moving their hands in the opposite direction as depicted on the computer monitor) and suppress the well-learned relationship between visual and motor coordination [34]. Participants in this study were instructed to accomplish a computerised activity comparable to oculomotor activity and reflector image diagrams that was designed in MATrix LABoratory (MATLAB) using the PsychToolbox [35, 36].  Figure 1 shows the MATrix LABoratory single-buffered drawing model.

Every session required participants to use a mouse to sketch the boundary of the given pictures, as shown in Figure 2. The mouse's left and right movements were reversed by the programme. The participants were requested to hold down the left mouse key during the tracing, and the tracing was discontinued when they let off of the key. Prior to signal data acquisition, all subjects were given 10 pretesting chance to acquaint themselves for predesigned assignment. Studied subjects were instructed to finish the reproduction or draw over in less than 300–360 seconds in every signal data acquisition test. All subjects were instructed to trace as precisely as possible within the boundary and to return to the border at the same point where the tracing left it. On a psychometric response scale for oculomotor activity of 1 to 7, participants were instructed to assess the complexity of the tracing, with 1 being “not difficult at all” and 7 representing “extremely tough.”

### 2.3. Data Collection

The draw over assignment and the single channel-EEG data acquisition were managed by two independent computers. Before each experiment, the clocks were synchronised. A 32″ liquid crystal display (LCD) display was used to show the sketching activity to the subjects, which was situated 30″ from their foreheads.

The MATLAB programme accumulated behavioural data such as timeframe (the time from the very first mouse pointer motion until the last observed motion), completion rate (the percentage of draw over activity which was accomplished by subjects), preciseness (the fraction of draw over activity that the studied participants prepared within the border of the displayed picture), and interpretive rating of task complexity along with the true tracing route. The NeuroSky Mind Wave Mobile headset was used to capture single-channel EEG data from the volunteers' foreheads at a frequency range of 480 Hz.

The Mind Wave Mobile headset is an EEG-monitoring device that safely detects brainwave patterns and tracks individuals' attention levels as they interact with various apps. It detects brain signals, filters out background noise and electrical interference, and transforms to digital power.

During the experiment, EEG data were wirelessly sent and recorded on the data gathering compute (Figure 3).

### 2.4. Practice and Evaluation of EEG Single

Real-time EEG data were captured at 512 Hz, and the frequencies within 0.5 and 45 Hz were recovered. The dataset was then subjected to a wavelet--based filter to eliminate eye blink and movement artefacts.

The eye-blinks and movement of the eye balls are a common difficulty encountered during the clinical recording of electroencephalogram (EEG) signals. Changes in the electric fields are around the eyes, and hence over the scalp, are caused by eye blinks. As a result, EEG recordings are frequently highly distorted, making interpretation difficult. Here, we applied a stationary wavelet transform (SWT) to the corrupted EEG to correct for the presence of the ocular artefact (OA) or movement artefacts (MA) [37].

The commencement and departure times of mouse pointer motion were used to fragment continuous EEG into epochs. For all preprocessed EEG segments, short-time Fourier transformations with 50 percent overlapping 2s hamming windows were calculated. Individual individuals' average power spectra were then calculated across segments for each trial they completed [35, 38].

The hamming window is a reduction created by a raised cosine with nonzero endpoints that is tailored to minimise the side lobe closest to it. It was suggested for smoothing the time domain truncated auto covariance function. The hamming window is most commonly seen in signal processing literature, where it is one of many windowing methods for smoothing values. It is also called as a tapering function or apodization (that indicates “removing the foot,” i.e., smoothing irregularities at the start and finish of the sampled signal).

The frequency band is depicted in Table 2.

## 3. Results

We have included 10 healthy control participants (7 male, 3 female) to match the remaining 10 depressive patients (7 male, 3 female) so that there was no considerable difference in age or sex between the two groups. All participants were passed through a sequences of investigation tests that measured perspicacity, ability of the visual system to distinguish objects from the background, and intellectual power to see whether there were any additional characteristics that could affect task performance. The Freiburg visual acuity and contrast test (FrACT) was used to assess the participants' visual acuity and contrast sensitivity at a distance of 200 cm [39]. The Sloan Letters have ten options, the Tumbling *E* has four, and the Landolt-C has four or eight. In a nutshell, 4 directions are less likely to be confused; however, the predicting probability is larger, necessitating more trials; 8 places allow for a faster determination of visual acuity (fewer trials) due to the lower predicting probability. The final result should be identical, but the number of runs must be carefully selected. Wilkinson [40] measured premorbid IQ, and researchers used the reading subtest of Othe wide range achievement test (WRAT). Exclusion criteria included incapability to demonstrate normal or corrected-to-normal vision (visual acuity score >1.0), inability to rectify low-contrast stimulation (2 percent contrast or less), as measured by a contrast sensitivity threshold score of >50, and a WRAT percentile score of less than 50%. Subjects who did not fit the above-mentioned diagnostic criteria were also eliminated from the study (Table 3).

The average rating for task completion difficulty rating for depression patients' and in control group is shown in Figure 4. And the trial completion time is shown in Figure 5. Trials 4,6, and 9 were the most challenging job for most participants, whereas Trials 3,7, and 10 were the.eEasiest, and others were considering under moderate category. The normalised perceived difficulty rating had 0.512, 0.623, and 0.821 correlations with the length of the pathway, the integer of inclination in the pathway, and the total duration to complete every test observed, respectively (*p* < 0.001), among depression patients. While the rating was 0.182, 0.236, and 0.382 that were reported among control group, and there was no statistical significance association reported between rating scale and time spent on each trial (*p*=1.43). The number of severe changes in path direction resembles to the integer of curves for the pathway reported by patients' group. The normalised perceived complexity and the mean frequency with which each participant finished each trial had no clear linear relationship. Tracing accuracy has also been proven to be independent to operating velocity and period in recent testing.

It can be seen that Figure 5 represents time spent on each trial by the studied participants. Overall, maximum time taken by patients' group is as follows: highest time was taken on task 4 (260 seconds), 6 (280 seconds), and 9 (290 seconds). In comparison with their counterparts (participants from the control group), for trials 4, 6, and 9, less time taken, 180 seconds, 190 seconds, and 200 seconds, respectively. *X*-axis denotes trails. *Y*-axis denotes task completion time in seconds in Figure 5. For both groups, Table 4 shows the relationship between average band power and each trial observation. The mean EEG power in the alpha-rhythm of upper cutoff, alpha- rhythm of lower cutoff, and beta-rhythm of lower bands of the complete experiment indicated a significantly reciprocal correlation with individual participants' experienced severity in the depressed patients' group, but no such relationship was seen in the power in other EEG bands. Drawing precision was completely irrelevant to EEG spectrum strengths at the frontal site throughout the study. Additionally, there was a considerable relationship between the upper and lower alpha band power (*p* < 0.01) and upper beta band power (*p* < 0.05) and a strong correlation between task performance accuracy and perceived problems.

The link among data gathered from distinct time-frame sections and total observed (incertitude) complexity was analysed, as indicated in Table 5, despite the fact that the power spectrum of the EEG changed throughout time intervals. While looking into the depressive disorder patients' group, the first 30 minutes in cooperation of theta-rhythm in frontal and alpha power rhythm showed significant associations with incertitude complexity of every task, but their relevance faded over time, especially theta power. While in the control group, no significant association in studied EEG characteristics was observed in the time frame. Only the first 30 seconds of each trial's EEG activity are indicative of the subjects' perceived difficulty during the visual-motor task; data obtained after that are likely due to other spatiotemporal variables introduced to the individuals or created through them.

Figure 6 shows the fraction modifications in mean power spectrum density compared to total average activity in the initial 30 seconds of the further challenging tests. The fourth test has greatest complexity. Test 5 was easier to complete apart from Tests 6 and 9. Trials 4 and 9 statistically have no effect on the average idiosyncratic difficulty grading for all tests in the experimentations.

## 4. Discussion

Detecting the variations in brain activity and movement that underpin mental illnesses is critical for better understanding the onset of these disorders and developing effective treatments. As a result, the researchers believe that more research into the brain's altered processing of visual information as a result of depression is required. It might be good to evaluate and expand the usage of perception tests as investigation techniques and prospective methods of diagnosing electronic data processing abnormalities in sufferer of the mental disorders. Perception tests, for instance, could be used like a supplement to other methods of evaluating the efficacy of various medications as the treatment continues. However, because the experiential changes remain modest and demonstrated specifically when matching among sets, depression cannot be recognised by assessing visual perception [41].

Taking averages across trials and then across people is standard in EEG data processing, but multidimensional characterisation of independent variability is rarely documented [42]. Feedback averaging presumes that variations between single trials are caused by Fnoisy sums of artefactual and/or task-independent EEG activity that can be simply averaged away to reveal single, fixed (real) brain interaction patterns in both time domain (ERP) and frequency domain (ERSP) evaluate. Examining EEG and other dynamic brain imaging data on a test-by-test basis appears to be an important step toward a deeper comprehension of electrical brain dynamics [43, 44].

In this paper, authors present a novel technique for characterising test-to-test changeability in the interval realm. The results of which recommend that in single-trial data, the activities of a spatially compressed setup of procedures with coarsely corresponding average dynamics demonstrate robust amplitude fluctuations and multiple dynamic approaches. This study discovered a substantial link among the spectral properties of single-channel frontal EEG and the task's mental effort requirements in normal control group and depressive disorder patients. According to the findings, a large increase in mental workload caused a constant escalation in EEG activities in the higher alpha band rhythm (between 11 and 14 Hz) in case of patients suffering from the depression.

Mental emotions can affect the EEG recorded from various parts of the brain. Negative feelings have been connected to brain waves in the right frontal lobe, while happy feelings have been connected to waves in the left frontal lobe [45, 46]. Asymmetry in brain electrical activity could indicate depression or the potential for depression. According to research, the right frontal cortex activity in depressed people is higher than the left frontal cortex activity [47]. Brzezicka et al. (2017) conducted research on controlled and depressed patients who completed a reasoning task and then underwent 5 minutes of electroencephalography recording, with the results showing that the frontal alpha asymmetry index in the depressed group was characterized by greater variance than in the control group [48].

In the first 30 seconds of each trial, the link between frontal EEG activity and mental effort is strong in case of the control group. While depressive participants' EEG features showed significant variation, other temporal events that occurred beyond the first 30 seconds may have influenced this outcome. Other temporal events that occurred beyond the first 30 seconds may have influenced this outcome.

Our findings also demonstrated that the frequency of acute particular movements in the trace, rather than the real time required to complete the line of work, influenced the mental exertion level associated with the activity. There has been a lot of research into the relationship between theta and alpha signals and difficult and effortful activities [12, 25, 39, 40, 49, 50]. Furthermore, during a high-load activity, Gevins and Smith discovered that frontal theta power increased whereas parietal alpha power decreased [25, 40]. According to our findings, both frontal theta and alpha power have positive associations with mental exertion. The alpha power disparity between our results and those of Gevins and Smith is most likely due to the recording locations, Fz and Pz.

From a practical perspective, visual contrast tests are a quick, easy, and noninvasive procedure that could be refined further to serve as biomarkers for aberrant visual information processing in depression. This discovery provided light on the prospect of adopting a user-friendly mobile EEG technology to assess mental workload in everyday life.

## 5. Conclusion

In conclusion, we have used some of the most regularly used EEG variables to demonstrate the EEG association of cognitive burden in a rather basic motor movement.

EEG asymmetry differences observed in depressive disorder patients' group in theta and alpha band showed significant associations with incertitude complexity of given tasks and reduced relative left frontal asymmetry exhibit during the oculomotor activity.

More complex encoding and feature extraction techniques are needed to improve the effectiveness of the algorithm. Further study employing longitudinal and cross-modal designs is needed to assess the reliability, accuracy, and responsiveness of this proposed technique for determining diagnostic contrast increment thresholds in depression and other mental diseases such as schizophrenia. Because of the nature and neuronal activation pattern distinctions between motor and cognitive tasks, a distinct set of EEG characteristics may be detected.

## Figures and Tables

**Figure 1:** MATrix LABoratory single-buffered drawing model.

**Figure 2:** Ten shapes depicted in the draw over activity. Test 1–5 (first line-from left to right) and second line 6–10 (from left to right).

**Figure 3:** Data collection workflow.

**Figure 4:** Average task completion difficulty ratings.

**Figure 5:** Average time taken to complete each trial.

**Figure 6:** Modifications in fraction power spectrum for the most difficult trials seen in the group of depressed patients.

**Table 1:** Beck depression inventory score (BDI).

Levels of depression as per beck depression inventory	Total score

These ups and downs are considered normal	1–10
Mild mood disturbance	11–16
Borderline clinical depression	17–20
Moderate depression	21–30
Severe depression	31–40
Extreme depression	Over 40

**Table 2:** Frequency band.

Type of band	Hz

Delta	Up to 4
Theta	4–8
Alpha	(i) Lower alpha 8–11 (ii) Upper alpha 11–14
Beta	(i) Lower beta 15–30 (ii) Upper alpha 31–36
Gamma	(i) Lower gamma 37–45 (ii) Upper gamma 46–50

**Table 3:** Demographic data for healthy control and depressive disorder groups.

	Depressive disorder patients	Control group	*p* value

Sex	Male -7, Female -3	Male -7, Female -3	1.00
Age of participants (years)	27.3 ± 2.8	28.3 ± 3.2	0.25
Perspicacity (twenty-twenty vision)	1.62 (0.51)	1.31 (0.36)	0.60
Visual perception	162.5 (56.7)	170.5 (47.6)	0.75
Wide range achievement test (WRAT) percentile	88.7 (12.1)	82.4 (11.7)	0.82
Beck depression inventory score	35.6 ± 3.7	18.5 ± 1.8	0.001

**Table 4:** Associations among mean frequency strengths and outcomes in every experiment test observed among patients' group and control group.

	Pearson correlation with mean frequency strengths			
Band	Idiosyncratic difficulties in depressive disorder patients' group	Idiosyncratic difficulties in control group	Performance accuracy in depressive disorder patients' group	Performance accuracy in control group

Delta	0.12	0.16	−0.0056	0.127
Theta	0.19	0.15	−0.0712	0.238
Lower alpha	0.11^*∗*^	0.18	0.0348^*∗*^	0.762
Upper alpha	0.08^*∗∗*^	0.12	−0.0176^*∗∗*^	0.487
Lower beta	0.05	0.018	0.0659	0.892
Upper beta	0.016^*∗*^	0.13	0.0521	0.592
Lower gamma	0.025	0.030	0.0439	0.490
Upper gamma	0.07	0.021	0.0287	0.703

^*∗*^ *p* < 0.05; ^*∗∗*^*p* < 0.01.

**Table 5:** Associations among participants' idiosyncratic difficulties and EEG characteristics in specific time structure among both groups.

EEG characteristics	Correlation with idiosyncratic difficulties			
	Depressive disorder patients' group		Control group	
	First 30 s	Last 30 s	First 30 s	Last 30 s

Delta	0.134	0.123	0.101	0.074
Theta	0.238^*∗*^	0.276^*∗*^	0.123	0.085
Lower alpha	0.324^*∗∗*^	0.389^*∗∗*^	0.125	0.032
Upper alpha	0.437^*∗∗*^	0.463^*∗∗*^	0.006	0.043
Lower beta	0.147	0.234	0.076	0.078
Upper beta	0.101	0.143	0.082	0.097
Lower gamma	0.187	0.189	0.043	0.054
Upper gamma	0.054	0.190	0.050	0.043

^*∗*^ *p* < 0.05; ^*∗∗*^*p* < 0.01.

## Data Availability

The data used to support the findings of this study can be obtained from the corresponding author upon request.
